RETRACTED

# Mechanism of Hyperbaric Oxygen Combined with Astaxanthin Mediating Keap1/Nrf2/HO-1 Pathway to Improve Exercise Fatigue in Mice

**DOI:** 10.1155/2022/6444747

**Published:** 2022-07-13

**Authors:** Zheng Zhang, Binghong Gao

**Affiliations:** ^1^School of Kinesiology, Shanghai University of Sport, Shanghai 200438, China; ^2^School of Physical Education and Sport Training, Shanghai University of Sport, Shanghai 200030, China

## Abstract

**Objective:**

This work aimed to explore the application and optimization of the electrophysiological monitoring system to real-time monitor the exercise-induced fatigue (EIF) animals and investigate the intervention mechanism of hyperbaric oxygen (HBO) combined with natural astaxanthin (NAX) on EIF.

**Methods:**

First, a system was constructed for acquisition, processing, and feature extraction of electrocardiograph (ECG) signal and surface electromyography (EMG) signal for EIF monitoring. The mice were randomly divided into a control group (CG), EIF group (EG), HBO treatment (HBO) group, and HBO combined with NAX treatment (HBO + NAX) group. The effect of the constructed system on classification recognition of EIF was analyzed. The levels of serum antioxidative stress indicators of mice in each group were detected, including malondialdehyde (MDA), catalase (CAT), superoxide dismutase (SOD), glutathione (GSH), glutathione-peroxidation (GSH-Px), and total antioxidant capacity (T-AOC). In addition, the mRNA and protein levels of Keap1/Nrf2/HO-1 pathway related genes in liver tissue were detected.

**Results:**

The results showed that the normalized least mean squares algorithm effectively removed the motion artifact interference of ECG signal and can clearly display the signal peak, and high-pass filtering and power frequency filtering effectively removed the motion and baseline drift interference of surface EMG signal. The recognition sensitivity, specificity, and accuracy of the EIF recognition model based on the long- and short-term memory network were 90.0%, 93.3%, and 92.5%, respectively. Compared with the CG, the characteristics of ECG signal and surface EMG signal of the mice in the EIF group changed greatly (*P* < 0.05); the serum MDA level was increased obviously; the CAT, SOD, GSH, GSH-Px, and T-AOC levels were observably reduced (*P* < 0.05); the expressions of Keap1 and HO-1 in the liver were reduced remarkably, while the expression of Nrf2 was increased notably (*P* < 0.05). Compared with the EIF group, the characteristics of ECG signal and surface EMG signal of the mice in the HBO and HBO + NAX groups were obviously improved (*P* < 0.05); the serum MDA level was significantly reduced; the CAT, SOD, GSH, GSH-Px, and T-AOC levels were greatly increased (*P* < 0.05); the expressions of Keap1 and HO-1 in the liver were greatly increased, while the expression of Nrf2 was decreased sharply (*P* < 0.05).

RETRACTED

**Conclusion:**

Therefore, the feature extraction and classification system of ECG signal combined with surface EMG signal could realize real-time monitoring of EIF status. HBO intervention could improve the body's ability to resist oxidative stress through the Keap1/Nrf2/HO-1 pathway and then improve the EIF state. In addition, the improvement effect of HBO + NAX was more obvious.

## 1. Introduction

With the improvement of national living standards in recent years, people have paid more and more attention to the improvement of physical fitness, so sports have become the main way of national fitness [1]. Moderate sports can prevent cardiovascular disease and other diseases by improving the function of the body's capillaries [2]. Before participating in major sports events, sports athletes need high-intensity and long-term sports training. With the gradual increase in sports intensity, the production of exercise-induced fatigue (EIF) often affects the normal immune system function of the human body [3]. Fatigue is caused by many reasons, such as excessive consumption of energy substances in the body, and accumulation of certain metabolites during muscle movement and contraction. At this time, the nerve cells in the brain will turn into an inhibited state, and the disturbance of water and salt metabolism in the body and the imbalance of the homeostasis of the internal environment will cause fatigue [4]. Therefore, exercise-induced fatigue is a comprehensive and complex process, which is related to many factors and physiological changes.

With the progress of exercise, the degree of fatigue of the human body will gradually deepen, and physiological signals such as electrocardiograph (ECG) will change accordingly [5]. Physiological signals are used as objective indicators to evaluate EIF status, and they are noninvasive, safe, and convenient [6]. Studies have confirmed that ECG signal, surface electromyography (EMG) signal, and electroencephalogram (EEG) signal can objectively reflect EIF status, while ECG and EMG signals can reflect changes in the state of the heart and muscles [7, 8]. However, these signals are often interfered by the human body and the environment during the acquisition process, which in turn affects the extraction of useful information from the signals. Machine learning has been widely used in pattern recognition, such as traditional decision tree (DT), support vector machine (SVM), and artificial neural networks (ANN) [9]. Because the traditional pattern recognition method will be affected by the validity of the input signal, the complexity of the calculation is increased, and the generalization ability of the model is also restricted. The emergence of deep neural network (DNN) effectively solves the shortcomings of pattern recognition, so it is used in the classification and recognition of physiological signals, which is expected to improve the efficiency of EIF status recognition [10, 11].

RETRACTED

Studies have also confirmed that exhaustive exercise will cause damage to the liver tissue of the body to a certain extent. After excessive exercise, the active oxygen and other substances and oxidative stress levels in the body are significantly increased [12, 13]. Therefore, improving the body's ability to resist oxidative stress is of great significance for preventing cardiovascular system damage after EIF. Hyperbaric oxygen (HBO) is a treatment method that can adjust the body's oxygen content and then play a protective effect on organs, and it has been proven to have excellent antifatigue effects [14]. Natural astaxanthin (NAX) is a kind of strong antioxidant, which has anti-free radical activity and lipid peroxidation [15]. NAX has the effects of antifatigue, anti-free radicals, and reducing oxidative damage [16]. Keap1/Nrf2/HO-1 belongs to the resist oxidative stress signaling pathway, which plays an important role in improving the body's ability to resist oxidative stress, anti-inflammatory response, and antiapoptosis [17]. Therefore, whether HBO combined with NAX intervention can improve the body damage caused by EIF through the Keap1/Nrf2/HO-1 signaling pathway remains to be explored.

Based on this, male Kunming mice were selected as the research objects to prepare a model of exercise fatigue and used the method of HBO combined with astaxanthin for intervention treatment. Secondly, the ECG and EMG signals of mice were collected, filtered, and processed by feature extraction, combined with deep neural network to construct a mathematical model for classification and identification of exercise fatigue, and the changes of physiological signal characteristics of mice were analyzed. Finally, the changes in the antioxidant stress status of the mice after the intervention treatment and the differences in the expression levels of genes related to the Keap1/Nrf2/HO-1 signaling pathway in the liver tissue were examined. This work hopes to provide a reference for the intelligent classification and identification of electrophysiological signals of exercise fatigue and to provide reference materials for in-depth understanding of the mechanism of exercise-induced fatigue and the search for improvement methods.

RETRACTED

## 2. Materials and Methods

### 2.1. Experiential Materials

Male mice were purchased from Changsheng Biotechnology Co., Ltd. NAX was purchased from BioAstin® Natural Astaxanthin. Malondialdehyde (MDA), catalase (CAT), superoxide dismutase (SOD), glutathione (GSH), glutathione-peroxidase (GSH-Px), and total antioxidant capacity (T-AOC) enzyme-linked immunosorbent assay (ELISA) kits were all purchased from Shanghai Enzyme United Biotechnology Co., Ltd. PrimeScript™ RT reagent Kit (Perfect Real Time) and TB Green® Premix Ex Taq™ II (Tli RNaseH Plus) were purchased from Takara; Trizol reagent and RIPA lysate were purchased from Thermo Fisher Scientific. Quinoline dicarboxylic acid (BCA) protein quantitative detection kit, electrochemical luminescence (ECL) detection kit, and polyvinylidene fluoride membrane (PVDF) were purchased from Shanghai Biyuntian Biotechnology Co., Ltd. Rabbit anti-human Keap1 monoclonal antibody, rabbit anti-human Nrf2 polyclonal antibody, rabbit anti-human HO-1 monoclonal antibody, rabbit anti-human *β*-actin antibody, and horseradish peroxidase-labeled mouse anti-rabbit IgG secondary antibodies were all purchased From Abcam.

### 2.2. Construction of EIF Mouse Model

According to the random number table, 40 male mice were randomly divided into a control group (CG), a EIF group (EG), a HBO treatment (HBO) group, and a HBO combined with NAX treatment (HBO + NAX) group, with 10 mice in each group. The average age of all experimental mice was 30.5 ± 2.3 days, and the average weight was 22.4 ± 3.6 g. This experiment strictly followed the “3R principles” (i.e., replacement, reduction, and refinement) for animal experiments, and the research had been approved by the Animal Protection Committee of our hospital.

Before preparation of the EIF mouse model, it was necessary to measure the body mass of the mice in each group except for the CG. According to 3% of body mass, the corresponding lead wire was loaded on the tail of the mouse and the mouse was placed in the Morris water maze with a water temperature of 28°C and a water depth of 25 cm to swim. It should be trained every day until the mouse was exhausted (showing that the head cannot be raised when it was submerged in the water for 10 seconds, and it cannot be turned over when it was pulled out and placed prone on a flat surface). It should be trained once a day for 28 days. After training, the mice in the EIF group were kept in cages separately. Mice in the HBO group and HBO + NAX group were placed in the HBO cabin immediately after the training. The pressure was set to 1.30 ATA, the oxygen concentration was greater than 90%, and the mice inhaled oxygen for 1 hour after they were stable. After the pressure was uniformly reduced to normal pressure, the mice were housed in separate cages. After HBO treatment, mice in the HBO + NAX group were given 100 mg/kg/d of NAX by gavage for 28 consecutive days (solution concentration = 2.5 mg/ml). The mice in the CG had no weight-bearing swimming training for 28 days.

RETRACTED

### 2.3. Design for the Real-Time Monitory System of EIF

The mouse ECG signal and surface EMG signal during sports were collected. The data processing software was adopted for filtering and feature extraction. Then, a mathematical model for EIF classification and recognition was constructed.

The ECG signal in the motion state is a weak current signal. Therefore, in order to ensure that an effective ECG signal can be collected, the original signal needs to be multistaged before A/D conversion. The frequency of ECG signal was mainly distributed between 0.1 and 100 Hz, and it was very susceptible to interference from electromyographic signals and power frequency signals. Thus, it was necessary to design a high signal-to-noise ratio circuit that can suppress signal interference, as shown in Figure 1. The effective surface EMG signal frequency was mainly distributed between 0 and 150 Hz, and this signal was also very susceptible to interference from surrounding environmental noise. Therefore, when the EMG signal was collected, it was necessary to carry out multistage amplification and filtering of the signal. The acquisition and processing of surface EMG signal is shown in Figure 2.

ECG signal is a weak bioelectric signal, the effective frequency band is mainly distributed between 0.05 and 100 Hz, and the energy spectrum is mainly distributed at 0.5∼20 Hz. Since ECG signal is susceptible to interference from electromyographic signals, power frequency signals, baseline drift, and motion artifacts, motion artifacts have the greatest impact on ECG signal [18]. Therefore, the focus of this work was to use adaptive filtering algorithms to suppress the motion artifact interference.

The adaptive filtering algorithm used in this work was the normalized least mean squares (NLMS) [19]. In the application process, the step factor was optimized by inputting the square Euclidean norm of *a*(*n*) into the adaptive filter, then the step factor can be defined as follows:

(1) $$\begin{array}{c} \lambda \left(n\right)=\frac{1}{\alpha +a^{T}a\left(n\right)}. \end{array}$$

In the above equation, *λ* was the step factor, *α* referred to the correction factor (0 < *α* < 1), and *a*^*T*^ was the transposition of *a*.

Based on this, the weight coefficient in the NLMS algorithm can be updated as follows: *ω*(*n* + 1) = *ω*(*n*) + *λ*(*n*)*e*(*n*)*A*(*n*), where *ω* was the weight and *e* referred to the error.

RETRACTED

The surface EMG signal shows strong regularity, but it is also a weak electrical signal. Therefore, the signal is amplified by the amplifier circuit AD620. At this time, the gain can be set as follows: *G*_*AD*620_=1+49.4*k*Ω/*R*_*G*_, where RG referred to a resistor. The power frequency filter circuit was mainly composed of two T-type networks, and the center frequency calculation equation was given as follows: *f*_*center*_=1/2*πRC*=49.6*Hz*, where *R* was a resistor and *C* was a capacitor. The surface EMG signal is mainly divided into time-domain and frequency-domain indicators for analysis. The time-domain indicators include root mean square (RMS), average rectified value (ARV), and integrated electromyographic value (IEMG) [20]. The calculation equation of each indicator is shown as follows:

(2) $$\begin{array}{c} \text{RMS}=\sqrt{\frac{\int_{t}^{T}\text{sEMG}{\left(t\right)}^{2}\text{d}t}{T}},\\ \text{ARV}=\frac{\int_{t}^{T}\left|\text{sEMG}\left(t\right)\right|\text{d}t}{T},\\ \text{IEMG}=\int_{t}^{T}\left|\text{sEMG}\left(t\right)\right|\text{d}t. \end{array}$$

Frequency domain indicators include mean power frequency (MPF) and median frequency (MF), which could be calculated with the following equations:

(3) $$\begin{array}{c} \text{MPF}=\frac{\int_{0}^{\infty }\text{fPSD}\left(f\right)\text{d}t}{\int_{0}^{\infty }\text{PSD}\left(f\right)\text{d}t}, \end{array}$$

(4) $$\begin{array}{c} MF=\frac{\int_{0}^{\infty }\text{PSD}\left(f\right)\text{d}t}{2}. \end{array}$$

In equations (3) and (4), PSD(f) was the power spectral density function of the surface EMG signal.

A mathematical model for EIF classification and recognition was constructed based on long short-term memory network (LSTM network). The key of the LSTM network is the state of the cell, which is mainly divided into input gate, output gate, and forget gate [21]. The basic structure of the model is shown in Figure 3.

The forget gate is mainly used to control whether the information in the cell state should be discarded. It was assumed that the input and the state of the hidden layer at the previous moment were *u*_*t*_ and *v*_*t*−1_, respectively, and the output value of the forgetting gate was Output_*t*_=*σ*(*ω*_*u*_*u*_*t*_+*ω*_*v*_*u*_*t*−1_+*b*). First, the nonlinear neural layer Tanh needed to obtain a temporary cell state based on the current input and the state of the hidden layer at the previous moment. Secondly, the part of the information was added in the forget gate to the temporary cell state to update the cell state. The updated cell state was expressed as Cell_*t*_=Output_*t*_ × Cell_*t*−1_+*i*_*t*_ × Tanh(*ω*_*u*_*u*_*t*_+*ω*_*v*_*u*_*t*−1_+*b*). Finally, the output gate was used to control the output of information.

RETRACTED

The mathematical model training process for EIF estimation constructed by the LSTM network is shown in Figure 4. The optimal weight was obtained through continuous iterative update, and the training of the model was completed after the output value meets the requirements.

### 2.4. ELISA Experiment

The serum samples were acquired from each group of mice to detect MDA, CAT, SOD, GSH, GSH-Px, and T-AOC using the ELISA method. All experimental operations were completed in accordance with the kit instructions. It should dilute the specific antibody globulin with coating buffer, add 0.3 mL of reagent to each well, and incubate overnight at 4°C. After removal of the coating solution, it was washed three times with washing buffer for 5 min each time. 0.2 mL of diluted antigen-containing sample was added to each well and incubated at 37°C for 1 hour. After removing the coating solution, the washing buffer was adopted to wash 3 times, with 5 min each time. 0.2 mL of diluted enzyme-labeled specific antibody solution was added to each well and incubated at 37°C for 1 h. After removing the coating solution, it was washed three times with washing buffer for 5 min each time. 0.2 mL of substrate was added to each well to incubate for 30 min at room temperature. After addition of the stop solution, a multifunctional microplate reader (BIO-TEK, USA) was adopted to detect the optical density (OD) value of each well.

### 2.5. Real-Time Fluorescence Quantitative PCR Experiment

Mice were sacrificed by dislocation. The liver tissues were taken, washed with precooled saline, cut into small pieces, and stored in a refrigerator at −80°C. A part of myocardial tissue was taken, added with liquid nitrogen solution, and ground thoroughly to extract the total ribonucleic acid (RNA) according to the Trizol reagent method. Reverse transcription of complementary deoxyribonucleic acid (cDNA) was carried out according to cDNA reverse transcription kit. The cDNA was used as template, and the relative expression levels of target genes Keap1, Nrf2, HO-1, and GAPDH were detected using the instructions of real-time fluorescent quantitative PCR detection kit. The quantitative primer information of each target gene is shown in Table 1. The reduced glyceraldehyde-phosphate dehydrogenase (GAPDH) gene was used as an internal reference, and the relative expression level of the target gene was calculated according to the 2^−∆∆CT^ method.

### 2.6. Western Blot

The mice were sacrificed by dislocation, and the liver tissues were taken. After the tissues were washed with precooled saline, an appropriate amount of RIPA lysate was added, and the mice were placed in an ice box for full grinding. After centrifugation at 12000 rpm for 10 min, the supernatant was taken, and the concentration of the extracted protein was detected according to the instructions of the BCA protein quantitative detection kit. The 10% separation gel was prepared for protein sodium dodecyl sulfate-polyacrylamide gel electrophoresis (SDS-PAGE). The target protein bands were cut and transferred to PVDF membranes and then placed in a blocking solution containing 5% skimmed milk powder for sealing treatment at room temperature for 2 h. Then, it should add the diluted rabbit anti-human Keap1 monoclonal antibody (1 : 1000), rabbit anti-human Nrf2 polyclonal antibody (1 : 500), rabbit anti-human HO-1 monoclonal antibody (1 : 1000), and rabbit anti-human *β* -actin antibody (1 : 1000) to incubate overnight in a refrigerator at 4°C. After washing, the horseradish peroxidase-labeled mouse anti-rabbit IgG secondary antibody (1 : 10000) was added to incubate at room temperature for 1 hour. It should follow the instructions of the ECL detection kit to develop the target protein band and take pictures in the gel imaging system. In addition, the ImageJ software was adopted to detect the gray value of the target gene band. With *β*-actin gene as a control, it could calculate the relative gray value of other target genes.

RETRACTED

### 2.7. Statistical Analysis

The SPSS 19.0 software was applied for statistical processing of experimental data. All experimental data were expressed as mean ± standard deviation (¯$\bar{\text{x}}$ ± SD), and one-way analysis of variance process was used to compare differences between groups. *P* < 0.05 meant that the difference was statistically significant.

## 3. Results

### 3.1. EIF Classification Model Test

The mouse ECG signal and surface EMG signal were pretreated, and the results are shown in Figure 5. It can be observed from Figures 5(a)–5(c) that the original ECG signal had the influence of motion artifacts. After filtering with the NLMS algorithm, the effect of the artifacts of the ECG signal can be significantly improved, and the peak position of the signal can be easily determined.

As illustrated in Figures 5(d)–5(f), the original surface EMG signal had interference from motion artifacts and baseline drift, and the interference was more serious. After high-pass filtering and power frequency filtering, the interference of motion and baseline drift can be obviously removed, and the waveform of the EMG signal can be better distinguished.

The number of hidden layers in the LSTM model was set to 1 and the number of neurons was set to 9 to perform the classification test of the model. The results are shown in Figures 6(a) and 6(b). It can be known from the confusion matrix in Figure 6(a) that the model had good recognition effects for different animal models, among which the recognition effect for CG, EG, and HBO + NAX animal models was the best, followed by the HBO group. The convergence of the error curve in Figure 6(b) revealed that as the number of iterations increased, the training and verification loss functions showed excellent convergence speeds and effects.

RETRACTED

The comparison results of the classification and recognition of different classification models (DT, KNN, SVM, and LSTM models) are shown in Figures 6(c) and 6(d).  Figure 6(c) shows that the recognition sensitivity (90.0%), specificity (93.3%), and accuracy (92.5%) of the LSTM model were higher than those of the DT (50.0%, 56.7%, and 55.0%), KNN (70.0%, 76.7%, and 75.0%), and SVM (80.0%, 86.7%, and 85.0%).  Figure 6(d) illustrates that as the number of iterations increased, the classification accuracy of each model reached the best around 30 iterations, and the classification accuracy of the LSTM model was the highest.

### 3.2. Effects of HBO and NAX on Physiological Indicators of EIF Mice

The differences in swimming exhaustion time and body mass of mice in each group were compared, and the results are shown in Figure 7.  Figure 7(a) illustrates that compared with the CG, the swimming exhaustion time of the mice in the EIF group and the HBO group was significantly shorter, and the difference was statistically great (*P* < 0.05). Compared with the EIF group, the swimming exhaustion time of mice in the HBO group and HBO + NAX group was significantly longer, showing statistically difference (*P* < 0.05). Compared with the HBO group, the swimming exhaustion time of mice in the HBO + NAX group was longer, and the difference was statistically visible (*P* < 0.05). There was no significant difference in swimming exhaustion time between the CG and HBO + NAX group (*P* > 0.05).

Figure 7(b) illustrates that with the increase of time, the body mass of mice in each group increased significantly. In the second week, compared with the CG, the body weight of the mice in the EIF group and the HBO group was significantly reduced, and the difference was statistically significant (*P* < 0.05). Compared with the EIF group, the body weight of mice in the HBO group and HBO + NAX group increased greatly, and the difference was statistically significant (*P* < 0.05). Compared with the HBO group, the body mass of the mice in the HBO + NAX group increased significantly, and the difference was statistically significant (*P* < 0.05). There was no significant difference in body weight between the CG and HBO + NAX group (*P* > 0.05).

RETRACTED

### 3.3. Effects of HBO and NAX on ECG and Surface EMG Signal Characteristics of EIF Mice

The differences between the ECG signal characteristics (heart rate and respiratory frequency indicators) and the surface EMG signal characteristics (time-domain and frequency-domain indicators) of the mice in each group were compared, and the results are shown in Figures 8 and 9.  Figure 8 illustrates that compared with the CG, the heart rate of the mice in the EG and the HBO group was obviously faster, and the respiratory rate was slower, showing statistically great difference (*P* < 0.05). Compared with the EG, the heart rate of the mice in the HBO group and the HBO + NAX group was significantly reduced, and the respiratory rate was significantly increased, showing statistically significant difference (*P* < 0.05). Compared with the HBO group, the heart rate of the mice in the HBO + NAX group was significantly reduced, and the respiratory rate was significantly increased, showing statistically significant difference (*P* < 0.05). There was no significant difference in heart rate and respiratory rate between the CG and the HBO + NAX group (*P* > 0.05).

The difference between the surface EMG signal indicators of the lateral femoral muscles of each group of mice was detected, and the results are shown in Figure 9. It can be known that compared with the CG, the ARV, IEMG, and RMS of the mice in the EG and the HBO group were significantly increased, and the MPF and MF were significantly reduced, with statistically great differences (*P* < 0.05). Compared with the EG, the ARV, IEMG, and RMS of the HBO group and HBO + NAX group mice were greatly reduced, the MPF and MF were sharply increased, and the difference was statistically visible (*P* < 0.05). Compared with the HBO group, ARV, IEMG, and RMS of HBO + NAX mice were significantly reduced, MPF and MF were significantly increased, and the difference was statistically significant (*P* < 0.05). There was no significant difference in ARV, IEMG, RMS, MPF, and MF between the CG and HBO + NAX group (*P* > 0.05).

### 3.4. The Effect of HBO Combined with NAX on the Level of Resist Oxidative Stress in EIF Mice

The difference in the resist oxidative stress indicators MDA, CAT, SOD, GSH, GSH-Px, and T-AOC in the serum of each group of mice was detected, and the results are shown in Figure 10. It illustrates that compared with the CG, the MDA level of the EG and the HBO group was significantly increased, while the levels of CAT, SOD, GSH, GSH-Px, and T-AOC were significantly reduced, and the difference was statistically significant (*P* < 0.05). Compared with the EG, the MDA level of mice in the HBO group and HBO-NAX group was significantly reduced, while the levels of CAT, SOD, GSH, GSH-Px, and T-AOC were significantly increased, and the difference was statistically significant (*P* < 0.05). Compared with the HBO group, the MDA level of mice in the HBO + NAX group was significantly reduced, while the levels of CAT, SOD, GSH, GSH-Px, and T-AOC were significantly increased, and the difference was statistically significant (*P* < 0.05). There was no significant difference in MDA, CAT, SOD, GSH, GSH-Px, and T-AOC between the CG and HBO + NAX group (*P* > 0.05).

RETRACTED

### 3.5. Effect of HBO Combined with NAX on Keap1, Nrf2, and HO-1 Expression in EIF Mice

The differences in the expressions of Keap1, Nrf2, and HO-1 mRNA in the liver tissue of each group of mice were detected, and the results are shown in Figure 11. Compared with the CG, the expressions of Keap1 and HO-1 in the EG and the HBO group were greatly reduced, while the expression of Nrf2 was significantly increased, and the differences were statistically significant (*P* < 0.05). Compared with the EG, the expressions of Keap1 and HO-1 in the HBO group and HBO + NAX group were significantly increased, while the expression of Nrf2 was significantly decreased, and the difference was statistically significant (*P* < 0.05). Compared with the HBO group, the expressions of Keap1 and HO-1 in the HBO + NAX group were remarkably increased, while the expression of Nrf2 was greatly decreased, and the difference was statistically remarkable (*P* < 0.05). There was no significant difference in the expression levels of Keap1, Nrf2, and HO-1 mRNA between the CG and the HBO + NAX group (*P* > 0.05).

The differences in the expressions of Keap1, Nrf2, and HO-1 protein in the liver tissue of each group of mice were detected, and the results are shown in Figure 12. Compared with the CG, the expressions of Keap1 and HO-1 in the EG and the HBO group were reduced, while the expression of Nrf2 was increased, and the differences were statistically significant (*P* < 0.05). Compared with the EG, the expressions of Keap1 and HO-1 in the HBO group and HBO + NAX group were increased, while the expression of Nrf2 was decreased, and the differences were statistically significant (*P* < 0.05). Compared with the HBO group, the expressions of Keap1 and HO-1 in the HBO-NAX group were increased, while the expression of Nrf2 was decreased, shown with significance (*P* < 0.05). There was no significant difference in the expressions of Keap1, Nrf2, and HO-1 mRNA between the CG and the HBO + NAX group (*P* > 0.05).

## 4. Discussion

Under normal physiological conditions, the body can automatically metabolize harmful substances such as lactic acid during exercise, which can reduce the exercise-induced oxidative stress and inflammation. That will not only reduce damage to the body, but also reduce the occurrence of certain diseases [22, 23]. With the increasing of exercise duration and intensity, the metabolic function of the body is disordered, and the effective substances produced by the body cannot be metabolized and accumulated, which in turn causes tissue damage and systemic inflammation [24]. In order to realize real-time monitoring of EIF, ECG and EMG signals were collected here to construct a mathematical model for EIF status classification and recognition. ECG signal can reflect the heart activity state of the body in real time, and EMG signal can reflect the activity state of muscles and nerves [25, 26]. However, both ECG and EMG signals are weak signals and are easily interfered by environmental factors. Signal acquisition is often affected by motion artifacts, baseline drift, and other signal interference [27]. Based on this, the NLMS algorithm was adopted to process the ECG signal motion artifacts, and the high-pass filtering and power frequency filtering were applied to filter the EMG signal. It was found that the processed ECG and EMG signal waveforms were clearer, which was helpful for the extraction of characteristic indicators. Analyzing the characteristics of the ECG and EMG signal of EIF mice revealed that the heart rate, respiratory frequency, RMS, ARV, IEMG, MPF, and MF changed greatly. In order to combine indicators for classification and recognition of EIF status, it is often necessary to use pattern recognition, machine learning, and deep learning methods for fusion analysis [28]. Here, a mathematical model for EIF status classification and recognition was constructed based on the LSTM model. It was found that the recognition sensitivity (90.0%), specificity (93.3%), and accuracy (92.5%) of the LSTM model were higher than those of the DT [29], KNN [30], and SVM [31]. It suggests that the LSTM model can utilize time series signals and has the characteristics of long-term learning. Therefore, the LSTM algorithm can realize feature extraction from physiological signals, which is similar to the research results of Wang et al. [32].

RETRACTED

With the deepening of EIF status, the levels of oxygen free radicals and reactive nitrogen in the body gradually increase, causing severe oxidative stress damage [33]. This work detected the changes of serum MDA, CAT, SOD, GSH, GSH-Px, and T-AOC levels in mice. MDA is a metabolite of lipid peroxides, which can be used to assess the degree of lipid peroxidation in the body [34]. CAT, SOD, GSH, GSH-Px, and T-AOC indicators can be used to assess the body's antioxidant capacity [35]. An EIF model was constructed using exhaustive swimming training. The results found that the level of MDA in the serum of the mouse was significantly increased, while the levels of CAT, SOD, GSH, GSH-Px, and T-AOC were significantly reduced. It shows that after EIF, the mouse body shows metabolic dysfunction and reduced antioxidant capacity [36]. Huang et al. [17] showed that the Keap1/Nrf2/HO-1 signaling pathway was involved in the regulation of anti-inflammatory and antioxidative stress responses [17]. Nrf2 is a key transcription factor in the Keap1/Nrf2/HO-1 signaling pathway, which can regulate the body's oxidative stress level [37]. Activating the Keap1/Nrf2/HO-1 signaling pathway can reduce the damage caused by the body's oxidative stress [38]. The results of this work found that the expressions of Keap1 and HO-1 in the liver tissue of EIF mice were reduced, while the expression of Nrf2 was increased. It showed that oxidative stress occurred after EIF, which in turn caused damage to the liver tissue of mice.

NAX shows a strong ability to resist oxidative stress, so it has a better protective effect on the liver [39]. HBO can play a protective effect on organs by increasing the body's oxygen content [40]. Therefore, NAX and HBO can be used to improve the damage state of organs after EIF. In this study, HBO and NAX were used for intervention treatment, and it was found that the level of MDA in the serum of mice was significantly reduced, while the levels of CAT, SOD, GSH, GSH-Px, and T-AOC were significantly increased, and the improvement effect of HBO combined with NAX was more obvious. In addition, compared with EIF mice, the expressions of Keap1 and HO-1 in mice after HBO and HBO combined with NAX treatment were significantly increased, while the expression of Nrf2 was significantly reduced. It is suggested that HBO and NAX intervention therapy can play a preventive effect on sports fatigue by regulating the physiological state of EIF mice, improving the body's resist oxidative stress level, and reducing liver tissue damage.

## 5. Conclusion

HBO could effectively increase the exercise time of exhausted mice by regulating the Keap1/Nrf2/HO-1 signaling pathway, regulate the physiological state of exercise, enhance the body's resist oxidative stress level, and protect the liver function of mice. Supplementing NAX on the basis of HBO intervention therapy showed a more excellent improvement effect. However, it only verified the effect of HBO combined with NAX in improving EIF status at the level of animal experiments, and the clinical efficacy of HBO combined with NAX had not been confirmed in this work. Therefore, in future studies, it is hoped that more samples will be included for the analysis of the clinical therapeutic effect of HBO combined with NAX in the treatment of EIF. The results could provide a basis for the prevention and treatment of sports fatigue and improve the effects of sports training.

RETRACTED

## Figures and Tables

**Figure 1:** Acquisition and processing of ECG signal.

**Figure 2:** Acquisition and processing of surface EMG signal.

**Figure 3:** The basic structure of LSTM.

**Figure 4:** Training process of the EIF classification model.

**Figure 5:** Preprocessing of ECG and EMG signals. Note: (a) the original ECG signal; (b) the ECG signal processed by the NLMS algorithm; (c) the ECG signal peak label after the processing; (d) the original surface EMG signal; (e) the surface EMG signal after high-pass filtering; and (f) the surface EMG signal after power frequency filtering.

**Figure 6:** Validation of EIF classification model. Note: (a) the confusion matrix; (b) the error convergence curve; (c) the recognition value comparison; and (d) the recognition accuracy.

**Figure 7:** Swimming exhaustion time and body mass changes of mice in each group. Note: (a) the swimming exhaustion time and (b) the weight change of each group. a, b, and c meant *P* < 0.05 compared to the CG, EG, and HBO groups, respectively.

**Figure 8:** Comparison of differences in ECG indicators of mice in each group. Note: (a) the comparison of heart rate and (b) the comparison of respiratory rate. a, b, and c meant *P* < 0.05 compared to the CG, EG, and HBO, respectively.

**Figure 9:** Comparison of differences in the surface EMG signal indicators of the lateral femoral muscle of mice in each group. Note: (a)–(e) the ARV, IEMG, RMS, MPF, and MF, respectively; a, b, and c meant *P* < 0.05 compared to the CG, EG, and HBO group, respectively.

**Figure 10:** Comparison of differences in serum resist oxidative stress indexes of mice in each group. Note: (a)–(f) meant MDA, CAT, SOD, GSH, GSH-Px, and T-AOC, respectively. a, b, and c meant *P* < 0.05 compared to the CG, EG, and HBO group, respectively.

**Figure 11:** Comparison of the expressions of Keap1, Nrf2, and HO-1 mRNA in the liver of mice in each group. Note: (a) the expression of Keap1; (b) the expression of Nrf2; and (c) the expression of HO-1; a, b, and c meant *P* < 0.05 compared to the CG, EG, and HBO group, respectively.

**Figure 12:** Comparison of the expressions of Keap1, Nrf2, and HO-1 protein in the liver of mice in each group. Note: (a) the Western blot detection results; (b) the expression of Keap1; (c) the expression of Nrf2; and (d) the expression of HO-1; a, b, and c meant *P* < 0.05 compared to the CG, EG, and HBO group, respectively.

RETRACTED

**Table 1:** Quantitative primer information of target gene.

Gene name	Primer sequence (5′ ⟶ 3′)	Size of product (bp)
Keap1	F: TCGAAGGCATCCACCCTAAG	135
	R: CTCGAACCACGCTGTCAATCT	
Nrf2	F: GGTCACGCTAATGCAGACAAT	223
	R: TCTTCTCAGGGGTATTCGCTTT	
HO-1	F: GATGGCGTCACTTCGTCA	118
	R: CCACTGGAGGAGCGGTGTC	
GAPDH	F: TGGCCTTCCGTGTTCCTAC	178
	R: GAGTTGCTGTTGAAGTCGCA	

## Data Availability

The data used to support the findings of this study are included within the article.
